# Osthole-Loaded Nanoemulsion Enhances Brain Target in the Treatment of Alzheimer's Disease via Intranasal Administration

**DOI:** 10.1155/2021/8844455

**Published:** 2021-01-25

**Authors:** Yilei Song, Xiangyu Wang, Xingrong Wang, Jianze Wang, Qiulian Hao, Jifu Hao, Xueqin Hou

**Affiliations:** ^1^College of Pharmacy, Shandong First Medical University & Shandong Academy of Medical Sciences, Taian, Shandong 271016, China; ^2^Institute of Pharmacology, Shandong First Medical University & Shandong Academy of Medical Sciences, Taian, Shandong 271016, China

## Abstract

Osthole (OST) is a natural coumarin compound that exerts multiple pharmacologic effects. However, the poor water solubility and the low oral absorption of OST limit its clinical application for the treatment of neurologic diseases. A suitable preparation needs to be tailored to evade these unfavourable properties of OST. In this study, an OST nanoemulsion (OST-NE) was fabricated according to the pseudoternary phase diagram method, which was generally used to optimize the prescription in light of the solubility of OST in surfactants and cosurfactants. The final composition of OST-NE was 3.6% of ethyl oleate as oil phase, 11.4% of the surfactant (polyethylene glycol ester of 15-hydroxystearic acid: polyoxyethylene 35 castor oil = 1 : 1), 3% of polyethylene glycol 400 as cosurfactant, and 82% of the aqueous phase. The pharmacokinetic study of OST-NE showed that the brain-targeting coefficient of OST was larger by the nasal route than that by the intravenous route. Moreover, OST-NE inhibited cell death, decreased the apoptosis-related proteins (Bax and caspase-3), and enhanced the activity of antioxidant enzymes (superoxide dismutase and glutathione) in L-glutamate-induced SH-SY5Y cells. OST-NE improved the spatial memory ability, increased the acetylcholine content in the cerebral cortex, and decreased the activity of acetylcholinesterase in the hippocampus of Alzheimer's disease model mice. In conclusion, this study indicates that the bioavailability of OST was improved by using the OST-NE via the nasal route. A low dose of OST-NE maintained the neuroprotective effects of OST, such as inhibiting apoptosis and oxidative stress and regulating the cholinergic system. Therefore, OST-NE can be used as a possible alternative to improve its bioavailability in the prevention and treatment of Alzheimer's disease.

## 1. Introduction

Alzheimer's disease (AD) is a common neurodegenerative disease characterized by memory impairment and cognitive dysfunction. The pathogenesis of AD is complex, including cholinergic dysfunction, oxidative stress, glutamate excitotoxicity, and amyloid *β* accumulation [1, 2]. To date, existing medications are symptomatic, and there are still no ideal therapeutic agents that can fundamentally cure AD [3].

Osthole (OST) is a natural coumarin compound extracted from the seed of *Cnidium monnieri* (L.) Cuss [4]. OST exerts various pharmacologic actions, such as anti-inflammation [5], antioxidative stress [6], antiapoptosis [7], and antitumor activities [8]. Many studies have disclosed that OST can prevent glutamate-induced neurotoxicity and neuronal loss and can be used to treat central nervous system disorders by modifying oxidative stress [9] and other molecular pathways [10–12]. In addition, OST also betters cognitive function and improves neuronal recovery [6, 13]. However, the poor water solubility and the low bioavailability [14, 15] hinder the clinical application of OST for the treatment of neurologic disorders. Furthermore, OST is pH-sensitive [16], which also affects its application. Generally, coumarin components are unstable to acids and prone to isoamyl double bond cracking. Although OST is also a natural coumarin compound, there is a pyranone ring with the property of unsaturated lactone, and the substituent in C7 position is methoxy structure in the molecular structure. The substituents in the C7 position increase the steric hindrance effect, thus improving its pH sensitivity for the drug.

Nanoemulsions are generally considered to be ideal drug carriers for the delivery of poorly water-soluble drugs to improve the bioavailabilities [17]. As a colloidal system, nanoemulsions are composed of oil, water, and a mixture of surfactants and cosurfactants [18]. The presence of oil and surfactants offers the highest drug solubilizing capability for hydrophobic drugs. The oil loaded with a drug is thoroughly dispersed into the water with the aid of surfactants and cosurfactants to form small droplets with a particle size in the nanometer range. Therefore, the solubility and bioavailability of poorly water-soluble drugs, such as OST, can be correspondingly enhanced due to the formation of nanoemulsions. Moreover, recent studies have shown neuroprotective effects were exerted by using naringenin nanoemulsion in the AD model [19] and in Parkinson's disease model [20], suggesting that nanoemulsion is a promising approach for developing new agents against neurodegenerative diseases.

The delivery of a drug to the brain via the oral route can be limited by the blood-brain barrier (BBB), resulting in unsatisfying bioavailability [2]. Thus, an alternative route via the nasal administration has emerged, since the nose-to-brain path can provide a direct brain-targeted delivery of drugs [2]. Moreover, nasal brain transport of nanocomposites has been reported to be an available strategy [21]. Therefore, the development of drug-loaded nanoemulsions via the nose-to-brain path may enhance the brain targeting of a drug and improve the bioavailability. For example, Bhattamisra et al. [22] reported that intranasal administration of rotigotine-loaded chitosan nanoparticles enhanced brain-targeting efficiency and drug bioavailability in rats. Other studies also showed that the application of nanoemulsion facilitated the delivery of donepezil and memantine (two approved drugs for treating AD) to the brain via the intranasal route [23, 24]. These studies suggest that nanotechnology is a potential approach to enhance the nose-to-brain delivery of drugs in the treatment of AD.

The aim of this study is to develop OST-loaded nanoemulsion that can be delivered via the nasal route and to investigate whether this strategy can improve the OST bioavailability to treat AD. Thus, the OST nanoemulsions (OST-NE) were tailored and the physicochemical properties were characterized. Then, the pharmacokinetic features of OST-NE via the intranasal (IN) and intravenous (IV) routes were comparatively investigated. Finally, the anti-AD effects of OST-NE were determined in L-glutamate-induced SH-SY5Y neuroblastoma cells and in scopolamine-induced AD mice.

## 2. Materials and Methods

### 2.1. Determination of Solubility and Lipid-Water Partition Coefficient of OST

Various types of oils, emulsifiers, and coemulsifiers were chosen as solvents to determine the saturated solubility of OST. Briefly, a number of OST powders (Nantong Feiyu Biological Technology Co., LTD., Nantong, China) were added to 0.5 mL of oils (ethyl oleate, isopropyl myristate), surfactant (polyethylene glycol ester of 15-hydroxystearic acid (HS-15), polyoxyethylene 35 castor oil (EL-35), Tween-80, the blended surfactant of HS-15 and EL-35 at a ratio of 1 : 1), and cosurfactant (polyethylene glycol 400 (PEG400), 1,2-propanediol, absolute ethanol), respectively. After stirring with a magnetic stirrer for 30 minutes, the mixture was shaken at 37°C for 48 hours and then centrifuged at 12000 r/min for 15 minutes. The supernatant was collected and diluted with methanol, and the content of OST was determined by high-performance liquid chromatography (HPLC) [25]. The chromatographic system consisted of a Shimadzu LC-10AT solvent delivery pump (Shimadzu, Kyoto, Japan) equipped with a 20 *μ*L loop and a UV visible detector. Welchrom C_18_ column (4.6 × 200 nm, 5 *μ*m) analytical column was used. The eluate was monitored at 322 nm. The mobile phase was methanol and water (80 : 20, *v*/*v*) with a flow speed of 1.0 mL/min at room temperature.

The lipid-water partition coefficient of OST was assayed with an octanol/water extraction method followed by HPLC analysis. Briefly, 40 mg of OST powder was dissolved in 2 mL distilled-water-saturated octanol in 5 mL polypropylene centrifugal tubes. Then, 2 mL of octanol-saturated distilled water was added into each tube. Each of the tubes was vibrated vigorously for 15 minutes and then shaken for 72 hours to reach equilibrium at 37°C. After centrifugation, the content of OST in the octanol and water was determined, respectively. The logarithm value of the lipid-water partition coefficient (log*P*) was calculated according to the following equation:

(1) $$\begin{array}{c} {}_{\log P=\log}\frac{C_{\text{oil}}\times V_{\text{oil}}}{C_{\text{water}}\times V_{\text{water}}}. \end{array}$$

### 2.2. Construction of Pseudoternary Phase Diagram

Pseudoternary phase diagrams were created using the aqueous titration method. The ratios of mixed surfactant to cosurfactant (Km values) were set as 1 : 1, 2 : 1, 3 : 1, and 4 : 1, respectively. The weight ratios of oil to the mixed surfactants at each Km were varied as 1 : 9, 2 : 8, 3 : 7, 4 : 6, 5 : 5, 6 : 4, 7 : 3, 8 : 2, and 9 : 1. After the oil and the mixed emulsifier were thoroughly merged, the mixture was titrated with distilled water under moderate stirring, and the amount of water was recorded when the transparent or translucent nanoemulsions appeared [26]. The pseudoternary phase diagrams were plotted according to the proportion of each component. Finally, the composition of OST-NE was 3.6% of ethyl oleate as oil phase, 11.4% of the surfactant (HS-15 and EL-35, ratio 1 : 1), 3% of PEG400 as cosurfactant, and 82% of the aqueous phase.

### 2.3. Physicochemical Characterization of OST-NE

Physical stability determination: OST-NE was centrifuged at 15000 r/min for 15 minutes. Whether OST-NE was precipitated, delaminated, or turbid after centrifugation was observed.

Particle size measurement: the zeta potential and particle size were determined by a Malvern Nano series particle size analyzer (Malvern, UK). The data analysis was performed using the Malvern Zetasizer software (Malvern, UK).

Type identification: the type of nanoemulsion was determined by using the oil dye Sudan Red III (red) and the water-soluble dye methylene blue (blue). The diffusion speed of the two dyes in the nanoemulsion was observed.

Morphological analysis: a drop of OST-NE was added on a carbon-coated copper grid and stained with 1% phosphotungstic acid. After drying, the morphology of the OST-NE was visualized using JEM-1200EX transmission electron microscopy (TEM) (JEOL, Tokyo, Japan).

### 2.4. Stability of OST-NE

The prepared OST-NE was placed at 25°C for 25 days. The particle size, polydispersity index (PDI), and potential of OST-NE were measured on 0, 5, 10, 15, 20, and 25 days.

### 2.5. Sterilization of OST-NE

To screen a proper sterilization method, OST-NE was sterilized by three sterilization methods, including high temperature autoclaving, ultraviolet (UV) irradiation, and microporous membrane. The stability of the OST-NE and bacteria in the OST was detected after sterilization.

### 2.6. *In Vitro* Drug Release Test

The OST-NE release test was performed using the intelligent dissolution test apparatus ZRS-8G (Tianjin Tianda Tianfa Technology Co., Ltd., Tianjin, China). The OST-NE or OST suspension (containing 4 mg OST) was placed in a dialysis bag (8000-14000 MW cutoff). The test was conducted in 200 mL of Simulated Nasal Electrolyte Solution (SNES) containing 1% Tween-80 at 100 r/min and 37 ± 0.5°C. The SNES (pH 5.5) was composed of 7.45 mg/mL NaCl, 1.29 mg/mL KCl, and 0.32 mg/mL CaCl_2_-2H_2_O. An aliquot (0.5 mL) of the dissolution medium was withdrawn at 0.25, 0.5, 1, 2, 4, 6, 8, 10, 12, 24, 36, 48, 60, and 72 hours, respectively. The dissolution medium was replenished with an equal volume of fresh isothermal SNES after each sampling. All the dissolution samples were filtered with a 0.22 *μ*m Millipore filter before analysis by HPLC.

### 2.7. Pharmacokinetic Study

Animal experiments throughout the study were approved by the Institutional Animal Ethics Committee of Shandong First Medical University and Shandong Academy of Medical Sciences. Kunming mice (20 ± 2 g) were purchased from the China Biologic Products Holdings, Inc. Mice were fed with a standard diet and had free access to distilled water. After fasting overnight, the mice were randomly divided into two groups. One group was administered with a single dose of OST-NE (40 mg/kg) by the IV route. Another group was administered with a single dose of OST-NE (10 mg/kg) by the IN route. Blood samples were collected through the orbital vein at 5, 15, 30, 60, 120, 180, 240, and 360 minutes after administration. Then, the mice were dislocated and perfused transcardially with normal saline. The brains were removed and homogenized in saline. The blood samples were centrifuged at 3000 r/min for 10 minutes. Then, 100 *μ*L of plasma or brain tissue homogenate was placed in a centrifuge tube, followed by adding 300 *μ*L acetonitrile. After being vortexed for 5 minutes, the samples were centrifuged at 10000 r/min for 10 minutes. The supernatant was collected. NaCl was added to the supernatant, and the sample was centrifuged at 10000 r/min for 10 minutes. The OST concentrations in the plasma and brain were measured using HPLC at 322 nm. DAS 2.2.1 software (DAS Studio, Shanghai, China) was used to calculate the pharmacokinetic parameters in plasma and brain tissue following IN and IV administration. To evaluate the brain targeting after IN administration, drug-targeting efficiency (DTE%) was calculated by formula (2), and drug-targeting percent (DTP%) [27] was calculated by formula (3).

(2) $$\begin{array}{c} \text{DTE}\%=\frac{\left[{\left({\text{AUC}}_{\text{brain}}/\text{AU}{\text{C}}_{\text{blood}}\right)}_{\text{i}.\text{n}.}\right]}{\left[{\left({\text{AUC}}_{\text{brain}}/\text{AU}{\text{C}}_{\text{blood}}\right)}_{\text{i}.\text{v}.}\right]}\times 100, \end{array}$$

(3) $$\begin{array}{c} \text{DTP}\%=\left[\frac{B_{\text{i}.\text{n}.}-B_{x}}{B_{\text{i}.\text{n}.}}\right]\times 100, \end{array}$$

(4) $$\begin{array}{c} B_{x}=\left(\frac{B_{\text{i}.\text{v}.}}{P_{\text{i}.\text{v}.}}\right)\times P_{\text{i}.\text{n}.}, \end{array}$$

where *P*_i.v._, *B*_i.v._, *P*_i.n._, and *B*_i.n._ denote the area under the curve (AUC) from time zero to time *t* (AUC_0−*t*_) of OST-NE in plasma (*P*) and brain (*B*) tissue that were obtained after IV and IN administration, respectively. *B*_*x*_ represents the brain AUC fraction contributed by systemic circulation through the blood-brain barrier (BBB) after IN administration.

### 2.8. Cell Culture and Treatments

The human neuroblastoma cell line SH-SY5Y was purchased from Capital Medical University (Beijing, China). SH-SY5Y cells were cultured with high-glucose Dulbecco's modified Eagle's medium (Hyclone, Logan, UT, USA) supplemented with 10% fetal bovine serum (EVERY GREEN, Zhejiang Tianhang Biotechnology Co., Ltd., Hangzhou, China) and 100 U/mL penicillin plus 100 *μ*g/mL streptomycin (Gibco, USA) at 37°C in a humidified 5% CO_2_ atmosphere in an incubator (WIGGENS, Germany).

To determine the condition of L-glutamate (L-Glu) in inducing excitotoxicity, SH-SY5Y cells were exposed to L-Glu (Solarbio Life Sciences, Beijing, China) at different concentrations (5, 10, 15, 20, 25, 30, 35, and 40 mmol/L) for different durations (4, 6, 8, 10, and 12 hours). MTT assay was used to determine the cell viability. Finally, an incubation of L-Glu at 30 mmol/L for 6 hours was chosen to establish the L-Glu-induced SH-SY5Y cell model.

Next, the effects of blank nanoemulsion on L-Glu-induced SH-SY5Y cells were investigated. SH-SY5Y cells were seeded in 96-well culture plates (2 × 10^4^ cells/well) and cultured for 24 hours. Then, the cells were treated with blank medium (model group) or blank nanoemulsion in medium (drug-free NE group, 10 *μ*mol/L and 0.1 *μ*mol/L) for 6 hours before exposed to 30 mmol/L L-Glu for another 6 hours. The control group was cultured with blank medium only. MTT assay was used to detect cell viability.

Then, the effects of OST-NE in L-Glu-induced SH-SY5Y cells were investigated. SH-SY5Y cells were seeded in 96-well culture plates (2 × 10^4^ cells, 100 *μ*L per well). After 24 hours of incubation, blank nanoemulsion (model), OST-NE (10 *μ*mol/L and 0.1 *μ*mol/L) were added and incubated for 6 hours. The culture medium was replaced by 30 mmol/L L-Glu in medium and incubated for 6 hours. The control group was cultured with blank nanoemulsion for 6 hours and then blank medium for 6 hours, respectively. MTT assay was used to detect cell viability.

### 2.9. Cell Viability Assay

The MTT assay was implemented as previously described [7]. After the aforementioned treatments, 20 *μ*L of MTT solution (5 mg/mL, KeyGEN BioTECH, Nanjing, China) was added to each well, and the plate was incubated at 37°C for 4 hours. The supernatant was discarded, 150 *μ*L of dimethyl sulfoxide was added to dissolve the formazan crystals, and the optical density (OD) was determined using a microplate reader (TECAN, Switzerland) at 570 nm [28]. The cell viability for each group was calculated by cell viability (%) = OD_experiment_/OD_control_∗100.

### 2.10. Terminal Deoxynucleotidyl Transferase- (TdT-) Mediated Deoxyuride-Triphosphate- (dUTP-) Biotin Nick-End Labeling (TUNEL) Staining

Apoptotic cells were detected by using the In Situ Cell Death Detection Kit (Roche) based on TUNEL technology. After OST-NE/L-Glu treatment, SH-SY5Y cells were fixed with 4% paraformaldehyde for 10 minutes and penetrated with 0.1% Triton X-100 for 1 minute at room temperature. The TdT and dUTP mixtures were added to the cells and incubated for 2 hours at 37°C. After three washes with phosphate-buffered saline, the cells were incubated with 4,6-diamino-2-phenylindole (DAPI) for 10 minutes at room temperature [11]. A fluorescence microscope (NIKON ECLIPSE C1, Japan) was used to capture images.

### 2.11. Biochemical Detection

Superoxide dismutase (SOD), malonaldehyde (MDA), glutathione (GSH), glutathione peroxidase (GSH-Px), and acetylcholine (Ach) (all kits were from Nanjing Jiancheng Bioengineering Institute, Nanjing, China) were measured according to the manufacturer's instructions. The activity of acetylcholinesterase (AchE) was detected according to the instructions of the enzyme-linked immunosorbent assay kit (Elabscience Biotechnology Co., Ltd., Wuhan, China). A microplate reader (TECAN, Switzerland) was used to detect the OD.

### 2.12. Western Blot Analysis

After treatment with or without OST-NE/L-Glu as described, SH-SY5Y cells from each group were collected, respectively. Total proteins were extracted with protein lysis buffer, and protein concentrations were determined using a BCA protein assay kit (Solarbio Life Sciences, Beijing, China). Proteins were separated by sodium dodecyl sulfate-polyacrylamide gel electrophoresis and transferred onto polyvinylidene fluoride membranes. After being blocked with 5% skim milk in tris-buffered saline containing 0.1% Tween-20 (TBST) for 1 hour, the membranes were incubated with primary antibodies at 4°C overnight: rabbit polyclonal anti-caspase-3 (1 : 500) (Servicebio, Wuhan, China), rabbit polyclonal anti-Bax (1 : 800) (Servicebio, Wuhan, China), and mouse polyclonal anti-*β*-actin (1 : 1000) (ZSGB-BIO, Beijing, China). Then, the membranes were washed three times with TBST, followed by incubating with horseradish peroxidase-conjugated anti-rabbit/mouse immunoglobulin G (IgG) antibody (ZSGB-BIO, Beijing, China) for 2 hours at room temperature. After three washes in TBST, the membranes were added with chemiluminescence solution and visualized via a gel imaging system. The images were analyzed using ImageJ software.

### 2.13. Learning and Memory Tests

Kunming mice (8-month-old) were randomly divided into five groups: vehicle, scopolamine, OST-NE (0.1 mg/kg), OST (25 mg/kg), and drug-free NE groups. The OST-NE (0.1 mg/kg) group was administered via IN, whereas the OST (25 mg/kg) group was administered intragastrically. The vehicle and scopolamine groups received the same amount of 0.9% saline intragastrically. The drug-free NE group received the same amount of blank nanoemulsion via IN. The frequency of administration was once daily for 21 days. On the 21st day, mice were intraperitoneally injected with 3 mg/kg scopolamine hydrobromide (Aladdin, Shanghai, China) 30 minutes after administration. Then, Morris water maze and light-dark box tests were performed according to our previous study [29]. Twelve hours after the behavioral experiments, blood was collected through the eyeball. The mice were euthanized and decapitated, and brain tissues were collected.

### 2.14. Statistical Analysis

The data are presented as the mean ± standard deviation (SD). The statistical analyses were performed using GraphPad Prism 6 software. Differences were analyzed using one-way analysis of variance (ANOVA). A *P* value less than 0.05 was defined as statistical significance.

## 3. Results

### 3.1. Solubilities of OST in Different Surfactants and Cosurfactants

Figure 1 shows the solubilities of OST in different surfactants and cosurfactants. The solubility of OST in ethyl oleate (37.03 ± 1.2 mg/mL) was higher than that in isopropyl myristate (27.1 ± 0.1 mg/mL). OST exhibited higher solubility in surfactants than in oils: HS-15 (180.6 ± 1.1 mg/mL), EL-35 (157.39 ± 7.6 mg/mL), Tween-80 (171.88 ± 8.1 mg/mL), and HS-15 and EL-35 (169.69 ± 8.1 mg/mL). In cosurfactants, the solubilities were 121.8 ± 8.9 mg/mL, 71.1 ± 5.8 mg/mL, and 9.8 ± 0.9 mg/mL in PEG400, absolute ethanol, and 1,2-propanediol, respectively.

### 3.2. Lipid-Water Partition Coefficient of OST

The concentrations of the two phases determined by HPLC were *C*_oil_ = 2.4 mg/mL and *C*_water_ = 1.4 *μ*g/mL, respectively. According to formula (1), log*P* was calculated to be 3.23.

### 3.3. Pseudoternary Phase Diagrams

The pseudoternary phase diagrams of different surfactants are shown in Figure 2. The shaded area was the largest when the surfactant was a mixture of HS-15 and EL-35 at a ratio of 1 : 1 and Km = 4 : 1 (Figure 2(c)).

### 3.4. Characteristics of OST-NE

The stability determination showed that the OST-NE was a clear, transparent, blue opalescent liquid with a slight odor before high-speed centrifugation. After centrifugation, the nanoemulsion was a light blue transparent liquid without delamination, turbidity, and precipitation. The average particle size of the OST-NE was 22.33 ± 0.47 nm, and the PDI was 0.115 ± 0.057 (Figure 3(a)). The particle size of OST-NE was small and uniform. The zeta potential of OST-NE was −9.88 ± 0.64 mv (Figure 3(b)). A type identification test showed that the diffusion rate of water-soluble dye methylene blue was faster than that of oil dye Sudan Red III (Figure 3(c)). The OST-NE particles were round in shape with a uniform size and good dispersion (Figure 3(d)).

### 3.5. Stability of OST-NE

As shown in Table 1, the particle size, PDI, and zeta potential of the OST-NE changed only slightly during storage, indicating that the prepared OST-NE had good thermodynamic stability.

### 3.6. *In Vitro* Release

The drug content of OST-NE in the dialysis bag was 4 mg, which was released in 200 mL of SNES release medium. The release of OST was increased in a time-dependent manner within 72 hours. However, the OST-NE released more OST than OST suspensions. By 72 hours, the OST-NE released approximately 80% of OST, whereas the OST suspensions only released about 40% of OST (Figure 4), indicating that the release rate of OST-NE in the body was relatively high. According to the principles of kinetics, the correlation between the cumulative release of OST and time was analyzed.  Table 2 shows the model fitting for the *in vitro* release profile of OST. The optimal mathematical model of the drug release process was explored by the value of the correlation coefficient *r* of the equation. The *in vitro* drug release process of OST-NE in SNES containing 1% Tween-80 conformed to the first-order kinetic model, and the OST suspension conformed to the Higuchi model.

### 3.7. Pharmacokinetic Profile

In plasma, the OST concentration reached the maximum just 5 minutes after administration by the IV route, whereas it took 30 minutes to reach the maximum concentration by the IN route (Figure 5). Moreover, the maximum concentration of OST in plasma by the IN route (3.53 ± 0.67 *μ*g/mL) was lower than that by the IV route (9.63 ± 1.44 *μ*g/mL). For AUC_0−*t*_ and AUC_0−∞_, there was no significant difference between IV and IN administration. The clearance rate by the IV route was 1.79 times higher than that of IN administration (Table 3).

In the brain, the maximum concentration of OST by IN (33.04 ± 2.56 *μ*g/mL, 5 minutes after administration) was higher than that by IV (25.62 ± 1.86 *μ*g/mL, 30 minutes after administration) (Figure 5 and Table 3). The AUC_0−*t*_ and AUC_0−∞_ of OST by IN were 0.61 times and 0.63 times higher than that of IV administration, respectively. The clearance rate by IV was 7.08 times higher than that of IN administration (Table 4).

The AUC_brain_/AUC_plasma_ values after IV and IN administrations of OST-NE were 2.82 and 4.88, respectively. The DTE% and DTP% of OST-NE after IN administration were 207.27% and 51.80%, respectively.

### 3.8. Sterilization Method of OST-NE

The OST-NE was layered after high temperature autoclaving (Figure 6(c)). Bacteria were still detectable in the OST-NE after 2 hours of UV irradiation, whereas no bacterium was detected by using a microporous membrane to sterilize. Therefore, the microporous membrane was used to filter the OST-NE.

### 3.9. Effects of OST-NE on the Activity of SH-SY5Y Cells

The neuroblastoma SH-SY5Y cell line is frequently chosen as a neuronal cell model in neurobiology [30–32]. In this study, SH-SY5Y cells were used to mimic AD as a cellular model and to assess whether OST-NE had a protective effect in this AD cellular model. To ensure the safety of OST-NE to the SH-SY5Y cells, the effects of OST-NE at different concentrations on the activity of SH-SY5Y cells were investigated. OST-NE at the concentration of 100, 50, and 25 *μ*mol/L significantly inhibited the viability of SH-SY5Y cells (19.97 ± 2.88%, 35.78 ± 4.72%, and 81.85 ± 12.09%, respectively), indicating that OST-NE at the concentration of over 25 *μ*mol/L was harmful to SH-SY5Y cells. While treated with 10 and 0.1 *μ*mol/L OST-NE, the cell viability changed insignificantly compared with the control group (Figure 7(a)), suggesting that 10 and 0.1 *μ*mol/L of OST-NE were safe for SH-SY5Y cells.

### 3.10. Effects of OST-NE on Cell Viability in L-Glu-Induced SH-SY5Y Cells

Glutamate overstimulation is associated with neuronal cell death [33] and may underlie the pathogenic mechanisms of AD [34]. L-Glu inhibited SH-SY5Y cells in a concentration-dependent manner in this study. The cell viability was decreased to 50% following incubation of L-Glu at 30 mmol/L for 6 hours (Figure 7(b)). Compared with the control group, the cell viability in the L-Glu group was significantly decreased (*P* < 0.01) (Figures 7(c) and 7(d)). After pretreating with blank nanoemulsion at 10 or 0.1 *μ*mol/L, the cell viability was altered insignificantly compared with the L-Glu group (Figure 7(c)). OST-NE of both doses (10 and 0.1 *μ*mol/L) increased the cell viability significantly compared with the L-Glu group (*P* < 0.01) (Figure 7(d)), suggesting that OST-NE had a protective effect.

### 3.11. OST-NE Protects SH-SY5Y Cells against L-Glu-Induced Apoptosis

TUNEL staining detects DNA damage by labeling the free 3′-hydroxyl termini [35]. During the early and late stages of apoptosis, genomic DNA breaks arise. So TUNEL staining is widely used as a measure of apoptosis, and TUNEL-positive cells are a specific parameter that indicates the apoptotic cells [36]. As shown in Figure 8, L-Glu treatment significantly increased the number of TUNEL-positive cells (red fluorescence-labeled cells) as compared with control SH-SY5Y cells, indicating that L-Glu (30 mmol/L) promoted the apoptosis of SH-SY5Y cells. Compared with the L-Glu group, the number of TUNEL-positive cells was decreased in the OST-NE pretreatment group, suggesting that OST-NE protected SH-SY5Y cells against L-Glu-induced apoptosis.

### 3.12. OST-NE Regulates Apoptosis-Related Proteins in L-Glu-Induced SH-SY5Y Cells

Bax and caspase-3 play important roles in the mechanisms of cell death in AD [37–39]. Bax is a proapoptotic effector [40], and caspase-3 is responsible for killing the cells at the end of the caspase cascades and mediates apoptosis [41]. L-Glu treatment significantly increased the relative expression of Bax and caspase-3 protein when compared with the control group (*P* < 0.05) (Figure 9). The relative expression of Bax and caspase-3 protein in the OST-NE pretreated group was lower than that in the L-Glu treated group (*P* < 0.05) (Figure 9), indicating that OST-NE inhibited the protein expression of Bax and caspase-3 induced by L-Glu.

### 3.13. OST-NE Increases Antioxidant Enzyme Activity in L-Glu-Induced SH-SY5Y Cells

Free radical-mediated oxidative damage may trigger the apoptosis and is also involved in the pathogenesis of AD [42]. Antioxidants are capable of inhibiting the radical chain reaction. Hence, they have great potential in the prevention and treatment of AD. SOD and GSH are two important endogenous antioxidants [43].  Figure 10 shows the activities of SOD and GSH in different groups. Both SOD and GSH activities were decreased in SH-SY5Y cells exposed to L-Glu compared with those of the control (both *P* < 0.05). OST-NE (0.1 *μ*mol/L) pretreatment increased the SOD and GSH activities significantly (both *P* < 0.01). OST-NE (10 *μ*mol/L) pretreatment also significantly increased the SOD activity (*P* < 0.01) and showed a trend to increase the GSH activity. These results indicate that OST-NE had antioxidative effects.

### 3.14. OST-NE Improves Learning and Memory Ability in Scopolamine-Induced AD Mice

In the Morris water maze test, the number of platform crossing in the scopolamine group was significantly decreased compared with the vehicle group (*P* < 0.05) (Figure 11(a)). The OST-NE group (0.1 mg/kg) and the OST group (25 mg/kg) showed higher number in crossing the platform than the scopolamine group. In the light-dark test, after a single electric shock training, the scopolamine group had the shortest step-through latency, indicating that the AD mouse model was successfully prepared. Compared with the scopolamine group, the step-through latency had a trend to be increased by IN administration of OST-NE (0.1 mg/kg) (Figure 11(b)). The difference between the drug-free NE group and the scopolamine group did not achieve statistical significance, suggesting that drug-free NE had little influence on the learning and memory ability.

### 3.15. OST-NE Regulates Oxidative Stress in Scopolamine-Induced AD Mice

SOD and GSH-Px are two major antioxidant enzymes, and MDA is an end product of lipid peroxidation. Thus, SOD, GSH-Px, and MDA were considered as markers for the evolution of oxidative stress in AD [42, 44]. Scopolamine caused a decrease in SOD activity (Figure 11(c)) and GSH-Px content (Figure 11(e)) and an increase in MDA content (Figure 11(d)), indicating that scopolamine induced oxidative damage. The SOD content in the OST-NE group was slightly higher than that in the scopolamine group (Figure 11(c)). The MDA content in the OST-NE group was lower than that in the scopolamine group (*P* < 0.05) (Figure 11(d)). Both OST-NE (0.1 mg/kg) and OST (25 mg/kg) increased the GSH-Px content compared with the scopolamine group (*P* < 0.05) (Figure 11(e)). SOD, GSH-Px, and MDA were altered very slightly with the treatment of drug-free NE when compared to the scopolamine group, suggesting that drug-free NE modulated the oxidative stress insignificantly.

### 3.16. OST-NE Regulates Cholinergic Pathway in Scopolamine-Induced AD Mice

Dysfunction of the cholinergic system is a key feature of AD, often characterized by altered Ach and AchE [45]. After treating with scopolamine, the Ach concentration in the brains of mice was significantly reduced (*P* < 0.05) (Figure 11(f)), whereas the activity of AchE was increased (*P* < 0.05) (Figure 11(g)), suggesting that scopolamine led to cholinergic system impairment. Compared with the scopolamine group, the Ach concentration in the cortex of the OST-NE group and the OST group was increased (*P* < 0.05) (Figure 11(f)), and the AchE activity in the hippocampus of the OST-NE group was significantly decreased (*P* < 0.05) (Figure 11(g)). There was no significant difference between the drug-free NE group and the scopolamine group. These results indicate that the cholinergic system may be regulated by OST-NE, but not by NE alone.

## 4. Discussion

To construct the OST-NE, the solubility of OST in different surfactants and cosurfactants was confirmed first. According to the solubility study, the solubility of OST in ethyl oleate was higher than that in isopropyl myristate (Figure 1). Therefore, ethyl oleate was selected as the oil phase. OST showed relatively high solubility in PEG400; hence, PEG400 was selected as the cosurfactant. In addition to water solubility, an optimal log*P* value is required for efficient uptake of a drug by cells [46]. This study showed that *C*_oil_ was greater than *C*_water_, and the log*P* was 3.23, indicating that OST had higher lipophilicity.

The shaded region in the pseudoternary phase diagram indicates the nanoemulsion domain; the larger the nanoemulsion region is, the stronger the emulsifying ability is [47]. The present study showed that the largest shaded area was when using a mixture of HS-15 and EL-35 (ratio 1 : 1) and when Km = 4 : 1 (Figure 2(c)). Compared with a single surfactant, the use of surfactant mixtures decreased droplet size and interfacial tension and showed higher storage stability in nanoemulsion [48]. Surfactant mixtures can reduce hydrophilic-lipophilic balance values, which enhances the lipophilic property of the surfactant blend and enhances the flexibility of surfactant layers that were formed [49]. Therefore, 11.4% of the HS-15 and EL-35 mixture was used as the surfactant, and 3.6% of ethyl oleate was used as the oil phase in the composition of OST-NE.

This study indicates that the OST-NE had good physical stability. Type identification suggests that the OST-NE was O/W type (Figure 3(c)). Smaller droplets have a greater interfacial area that significantly enhances the release rate of the drug [50]. The particle size of OST-NE was small and uniform, with an average particle size of 22.33 ± 0.47 nm. After being prepared into a nanoemulsion, the dissolution rate of OST can be significantly improved. Therefore, OST-NE released more OST than OST suspensions.

The AUC_brain_/AUC_plasma_ ratio represents the brain targeting coefficient of the drug. The AUC_brain_/AUC_plasma_ value after IV administration was lower than that by nasal administration of OST-NE. This indicates that OST-NE enhanced brain target by the IN route. The DTP% was greater than 50% by IN administration of OST-NE, indicating that half of the OST in the brain tissue entered the brain directly from the nasal cavity. It is known that drug absorption from the nasal cavity to the brain usually occurs through two pathways: (1) systemic pathway: a certain amount of the drug directly enters the systemic circulation and reaches the brain through the BBB; and (2) olfactory pathway: the drug enters the cerebrospinal fluid or brain directly from the nasal cavity [51]. DTE% and DTP% correspond to the percentage of drugs that are transported directly to the brain via the olfactory pathway. The higher DTE% and DTP% values imply that OST-NE had superior brain targeting efficiency. The drug can be quickly transported to the brain by IN administration, which may be due to the smaller particle size with improved transcellular transport [52].

Apoptosis is considered to be an important mechanism of AD [39]. Excessive L-Glu not only results in excitotoxicity but also induces cell death, which may underlie the AD neuropathology [53, 54]. Therefore, the L-Glu-induced cell model was used to investigate the effects of OST-NE on neuronal cell death. Consistent with other study [54], L-Glu at high concentrations significantly increased cell death by using the cell viability test and TUNEL analysis. It has been reported that OST has antiapoptotic activity [7]. In this study, OST-NE also protected the SH-SY5Y cells against apoptosis, suggesting that OST-NE remained the antiapoptosis activity of OST. The apoptosis pathway involves many modulators, including Bax and caspase-3. AD patients exhibited high expression of Bax [55] and an increase in procaspase-3 and active caspase-3 expression [38], indicating that Bax and caspase-3 are implicated in AD. Furthermore, Bax promotes the loss of mitochondrial membrane potential and the release of cytochrome c to the cytoplasm, resulting in the subsequent cleavage and activation of the apoptotic caspase-3 [56], suggesting Bax is an upstream modulator that triggers the activation of caspase-3 and apoptosis. Therefore, to further confirm the antiapoptotic effect of OST-NE, Bax and caspase-3 were determined. L-Glu increased the expression of Bax and caspase-3, which was consistent with other studies [57, 58]. OST-NE reversed the increased expression of Bax and caspase-3 induced by L-Glu. These results suggest that OST may prevent L-Glu-induced apoptosis by regulating apoptotic signals.

Oxidative stress is another key pathogenesis of AD [43]. Oxidative stress increases neuronal cell damage and apoptosis, leading to cognitive impairment [42]. SOD, GSH, and GSH-Px belong to the antioxidant enzyme system. In AD patients, the MDA level in the blood was higher along with a decrease in GSH levels, indicating elevated oxidative stress in AD [59]. SOD is a major component of the antioxidant system and limits the cytotoxic effects of toxic free radicals [60]. Similar to other study [61], L-Glu induced SOD activity reduction. OST-NE pretreatment significantly increased the activity of SOD and GSH, suggesting that OST-NE may protect SH-SY5Y cells from L-Glu-induced neurotoxicity by reducing oxidative stress. Furthermore, a scopolamine-induced mouse model of AD was employed to confirm the antioxidative effect of OST-NE *in vivo*, since scopolamine was able to decrease the activity of SOD and increase MDA in the brain [62]. Similar to the *in vitro* study, OST-NE treatment increased the level of SOD and GSH-Px in the serum. MDA is the final product of lipid peroxidation after biological membranes are attacked by reactive oxygen species. The level of MDA can reflect the degree of oxidative stress [63]. This study showed that the MDA level in the serum was significantly decreased in mice treated with OST-NE. Together, these results suggest the antioxidative effect of OST-NE.

Scopolamine not only causes oxidative stress but also impairs the cholinergic function and results in cognition dysfunction [62, 64]. In this study, scopolamine injection also impaired the learning and memory ability, reduced Ach level, and increased the AchE activity in mice. After administration with OST-NE via the nasal route in scopolamine-induced AD mice, the number of platform crossings was increased, indicating that OST-NE could improve the learning and memory. Cholinergic neurons located in the basal forebrain are severely lost in AD [65]. Ach is an important neurotransmitter in the central nervous system. Cholinergic neurons release Ach, which is hydrolyzed by the enzyme AchE. Loss of cholinergic neurons leads to reduction in Ach, further resulting in memory impairment in patients with AD [45]. OST-NE treatment increased the level of Ach and decreased the activity of AchE in the brain in AD model mice, indicating that OST-NE may be a potential agent for treating AD by regulating the cholinergic system.

## 5. Conclusion

By using nanoemulsion technology, a formulation of OST-NE was developed and was proved to be well targeted to the brain by the nasal route. Furthermore, OST-NE at a low dose exerts a protective effect on L-Glu-induced neurotoxicity and improves learning and memory in AD mice, which may be through regulating the apoptosis pathway, oxidative stress, and the cholinergic system. These findings suggest that OST-NE can be used as a possible alternative to improve its bioavailability and that OST-NE may have a potential curative effect in the prevention and treatment of AD.

## Figures and Tables

**Figure 1:** Solubility of OST in different surfactants and cosurfactants.

**Figure 2:** Pseudoternary phase diagrams of the oil-surfactant-water systems. The shaded region represents nanoemulsion. (a) EL-35 as surfactant; (b) HS-15 as surfactant; (c) a mixture of EL-35 and HS-15 at a ratio of 1 : 1 as surfactant; (d) Tween-80 as surfactant.

**Figure 3:** Characteristics of OST-NE. (a) Particle size of OST-NE. (b) Zeta potential of OST-NE. (c) The different diffusion velocity of oil dye Sudan Red III (left) and water-soluble dye methylene blue (right) in the OST-NE. (d) TEM images of OST-NE, scale bars = 500 nm (top left), 200 nm (top right), and 100 nm (bottom).

**Figure 4:** *In vitro* release of OST from nanoemulsion compared with suspension.

**Figure 5:** Pharmacokinetics curve of OST-NE in plasma and brain tissue after IN and IV administrations: (a) drug concentration in plasma; (b) drug concentration in the brain.

**Figure 6:** Influence of three different sterilization methods on the stability of OST-NE: (a) microporous filter; (b) UV sterilization; (c) autoclave.

**Figure 7:** Effect of OST-NE on cell viability in L-Glu-induced SH-SY5Y cells. (a) Effect of OST-NE on SH-SY5Y cell viability. *n* = 5‐8 per group, ^∗∗^*P* < 0.01 vs. control group. (b) Effect of L-Glu on the survival of SH-SY5Y cells. (c) Effect of blank nanoemulsion (drug-free NE) on cell viability in L-Glu-induced SH-SY5Y cells. *n* = 5‐8 per group, ^##^*P* < 0.01 vs. control group. (d) Effect of OST-NE on cell viability in L-Glu-induced SH-SY5Y cells. *n* = 6‐8 per group, ^##^*P* < 0.01 vs. control group, ^∗∗^*P* < 0.01 vs. model group.

**Figure 8:** Effect of OST-NE on L-Glu-induced apoptosis in SH-SY5Y cells by TUNEL staining: (a) control, (b) model (blank nanoemulsion+30 mmol/L L-Glu), (c) OST-NE (10 *μ*mol/L)+L-Glu (30 mmol/L), (d) OST-NE (0.1 *μ*mol/L)+L-Glu (30 mmol/L). Red: TUNEL-positive; blue: DAPI, scale bar = 50 *μ*m.

**Figure 9:** Effects of OST-NE on the protein levels of Bax and caspase-3 in L-Glu-treated SH-SY5Y cells. (a) Representative bands of Bax, caspase-3, and *β*-actin by Western blot analysis. (b) Relative protein levels were quantified by densitometry and normalized relative to the expression of *β*-actin. *n* = 3‐4 per group, ^##^*P* < 0.01 vs. control group, ^∗^*P* < 0.01 and ^∗∗^*P* < 0.01 vs. model group.

**Figure 10:** Effect of OST-NE on L-Glu-induced oxidative stress in SH-SY5Y cells. (a) GSH activity, (b) SOD activity. *n* = 3 per group, ^#^*P* < 0.05 vs. control group, ^∗∗^*P* < 0.01 vs. model group.

**Figure 11:** Effects of OST-NE on memory function, oxidative stress, and cholinergic pathway in scopolamine-induced mice. (a) The number crossing the platform during the space exploration in the Morris water maze test. (b) Latency to step to the dark chamber in the light and dark box test. (c–e) Levels of oxidative stress markers (SOD, MDA, and GSH-Px) in the serum. (f) Ach level in the cerebral cortex. (g) AchE level in the hippocampus. (a, b) *n* = 10‐12 per group, (c–g) *n* = 5‐6 per group. ^#^*P* < 0.05 and ^##^*P* < 0.01 vs. vehicle group, ^∗^*P* < 0.05 and ^∗∗^*P* < 0.01 vs. scopolamine group. Drug-free NE, blank nanoemulsion.

**Table 1:** Average particle size, PDI, and absolute zeta potential of OST-NE during storage.

Time (days)	Particle size (nm)	PDI	Zeta (mv)
0	21.09 ± 0.06	0.053 ± 0.013	−7.24 ± 1.85
5	21.22 ± 0.23	0.068 ± 0.014	−6.45 ± 1.90
10	21.61 ± 0.42	0.145 ± 0.032	−8.69 ± 2.12
15	21.12 ± 0.11	0.081 ± 0.006	−6.30 ± 3.66
20	20.96 ± 0.23	0.063 ± 0.002	−4.04 ± 1.10
25	22.16 ± 0.28	0.136 ± 0.015	−4.81 ± 1.06

**Table 2:** Model fitting for *in vitro* release profile of OST.

Model	Osthole nanoemulsion	*r*	Osthole suspension	*r*
Zero-order	*Q* = 1.2205*t* + 5.1462	0.9831	*Q* = 0.6085*t* + 3.3968	0.9804
First-order	Ln(100 − *Q*) = −0.0247*t* + 4.6188	0.9978	Ln(100 − *Q*) = −0.0079*t* + 4.5777	0.9904
Higuchi	*Q* = 11.084*t*^1/2^ − 10.955	0.9928	*Q* = 5.544*t*^1/2^ − 4.6974	0.9933

**Table 3:** Pharmacokinetic parameters of OST-NE in plasma after IN and IV administrations.

Parameters	*C*_max_ (*μ*g/mL)	AUC_0−*t*_ (*μ*g/mL∗h)	AUC_0−∞_ (*μ*g/mL∗h)	CL (l/H/kg)	MRT_0−*t*_ (h)
Intranasal	3.53 ± 0.67	2.90 ± 0.18	2.93 ± 0.22	2.86 ± 1.04	1.23 ± 0.30
Intravenous	9.63 ± 1.44	3.70 ± 0.51	3.74 ± 0.53	7.99 ± 0.69	0.52 ± 0.22

Note: *C*_max_: maximum concentration; CL: plasma clearance; MRT: mean residence time.

**Table 4:** Pharmacokinetic parameters of OST-NE in the brain after IN and IV administrations.

Parameters	*C*_max_ (*μ*g/mL)	AUC_0−*t*_ (*μ*g/mL∗h)	AUC_0−∞_ (*μ*g/mL∗h)	CL (l/H/kg)	MRT_0−*t*_ (h)
Intranasal	33.04 ± 2.56	16.87 ± 2.35	17.55 ± 2.48	0.36 ± 0.23	0.82 ± 0.14
Intravenous	25.62 ± 1.86	10.45 ± 2.69	10.80 ± 2.72	2.91 ± 0.54	0.47 ± 0.24

## Data Availability

The data are available from the corresponding author upon request.
